RETRACTED

# PATZ1 induces PP4R2 to form a negative feedback loop on IKK/NF-κB signaling in lung cancer

**DOI:** 10.18632/oncotarget.10427

**Published:** 2016-07-06

**Authors:** Ming-Yi Ho, Chi-Ming Liang, Shu-Mei Liang

**Affiliations:** ^1^ Genomics Research Center, Academia Sinica, Taipei 11529, Taiwan, ROC; ^2^ Agricultural Biotechnology Research Center, Academia Sinica, Taipei 11529, Taiwan, ROC

**Keywords:** epithelial-mesenchymal transition (EMT), IκB kinase (IKK), migration/invasion/metastasis, PATZ1, protein phosphatase 4 (PP4)

## Abstract

Activation of IKK enhances NF-κB signaling to facilitate cancer cell migration, invasion and metastasis. Here, we uncover the existence of a negative feedback loop of IKK. The transcription factor PATZ1 induces protein phosphatase-4 (PP4) regulatory subunit 2 (PP4R2) in an IKK-dependent manner. PP4R2 enhances the binding of PP4 to phosphorylated IKK to inactivate IKK/NF-κB signaling during sustained stimulation by cellular stimuli such as growth factors and inflammatory mediators. Matched pair studies reveal that primary lung cancers express more PATZ1 and PP4R2 than lymph node metastases in patients. Ectopic PATZ1 decreases invasion/colonization of lung cancers and prolongs the survival of xenograft mice. These effects of PATZ1 are reversed by downregulating PP4R2. Our results suggest that PATZ1 and PP4R2 provide negative feedback on IKK/NF-κB signaling to prevent cancer cells from over-stimulation from cellular stimuli; a decline in PATZ1 and PP4R2 is functionally associated with cancer migration/invasion and agents enhancing PATZ1 and PP4R2 are worth exploring to prevent invasion/metastasis of lung cancers.

## INTRODUCTION

Growth factors, inflammatory cytokines, pathogens and cellular stresses enhance NF-κB activity that regulates many target genes resulting in a variety of cellular responses [1]. NF-κB activity is inhibited by the binding of IκB which masks the nuclear localization sequence of NF-κB to modulate its regulation of downstream genes [2]. The inhibitory effect of IκB on NF-κB is in turn suppressed by the phosphorylated IκB kinase (phospho-IKK) that phosphorylates IκB to increase polyubiquitination and degradation of IκB [3]. Constitutive, aberrant elevation of active NF-κB is associated with chronic inflammatory diseases and many types of cancer [4].

Stimulation of lung cancer cells with growth factors and inflammatory mediators such as PGE2 increased the level of PIP3 to reach a plateau at 1 h and then declined [5]. This transient increase in PIP3 was accompanied by an increase in phosphorylated Akt and prohibitin (phospho-Akt^S473^ and phospho-PHB^T258^) resulting in transient upregulation of phosphorylation of IKK and NF-κB p65 [5]. The PGE2-mediated increase of phospho-Akt^S473^ dissipates within 2 h and reappears late after 12 h [6]. The resurgence of phospho-Akt^S473^ is due to migration-inducing factor 7 (MIG-7)-mediated inactivation of protein phosphatase 2A (PP2A) [6]. It is not clear, however, whether this resurgence of phospho-Akt^S473^ is also accompanied by an increase in phosphorylated IKK and NF-κB p65.

RETRACTED

Phosphorylation and dephosphorylation of signal mediators or effectors such as Akt, IKK and NF-κB by kinases and phosphatases serve as a reversible mechanism to switch on and off stimuli-mediated cellular processes like metabolism, apoptosis, proliferation and migration [5, 7]. The majority of oncogenes encode kinases to facilitate phosphorylation of signal mediators, whereas phosphatases such as PP2A primarily suppress phosphorylation of signal mediators or effectors to serve as cancer suppressors [8–10]. To monitor cellular activities, it is important to examine not only how quickly a signal mediator or effector such as Akt, IKK or NF-κB p65 has been phosphorylated and activated but also how long they remain in the activated (phosphorylated) state.

In this study, we found that even though phospho-Akt^S473^ in lung cancer cells reappeared 12 h after PGE2 or growth factor stimulation, this resurgence of phospho-Akt^S473^ was not accompanied by an increase in phosphorylated IKK and NF-κB p65. IKK and NF-κB p65 were sustained in the dephosphorylated state due to PP4. We also found that the increase in the effect of PP4 was primarily due to the increase in PP4 regulatory subunit 2 (PP4R2) that enhances the association of phospho-IKKα/β^S176/180^ with PP4 catalytic unit (PP4C) leading to dephosphorylation of phospho-IKKα/β^S176/180^. Additional studies revealed that the induction of PP4R2 was primarily due to a transcription factor, namely POZ/BTB and AT-hook-containing zinc finger protein 1 variant 4 (PATZ1) [11, 12]. The biological impact of PATZ1and PP4R2/PP4C negative feedback on IKK/NF-κB was further elucidated by upregulating and downregulating PATZ1 and PP4R2 to study their influence on the cellular effects of growth factors, PGE2 and PIP3 and the migration/invasion and colonization/metastasis of lung cancer cells *in vitro* and *in vivo*.

## RESULTS

### Homeostasis of IKK/NF-κB signaling

Stimulation of lung cancer cells with PGE2 or growth factors (EGF, HGF, IGF-1) results in transient increase of phospho-Akt^S473^, phospho-IKKα/β^S176/180^ and phospho-NF-κB p65^S536^ in the early phase (within 1 h) [5]. As the increase of phospho-Akt^S473^ has been shown to dissipate within 2 h and reappear in the late phase (about 12-48 h later) [6], we examined whether phospho-IKKα/β^S176/180^ and phospho-NF-κB p65^S536^ in lung cancer cells could be increased along with phospho-Akt^S473^ during the late phase of PGE2 stimulation. Our results showed that neither phospho-IKKα/β^S176/180^ nor phospho-NF-κB p65^S536^ was increased during the late phase (Figure 1A). Since phospho-IKKα/β^S176/180^ and phospho-NF-κB p65^S536^ may increase cellular COX-2 and epithelial-mesenchymal transition (EMT) [13], we analyzed the levels of COX-2, vimentin and E-cadherin transcription suppressors, notably Snail, ZEB-1 and Twist during the late phase. We found that the levels of ZEB-1 reached a plateau at 24-25 h and stayed at a relatively high level for a much longer time (> 17 h; Figure 1B). The level of Twist which is known to be increased by phospho-Akt-induced MIG-7 [6], was elevated at 27 h and remained at high level in the late phase (Figure 1B). In comparison, the levels of COX-2 and Snail peaked at 24-25 h and then decreased to the basal level 11 h later (Figure 1B), suggesting that they might be IKK/NF-κB dependent. Similar results were not only found in PGE2-treated (Figure 1) but also PIP3- and growth factor-treated lung cancer cells (Supplementary Figure S1).

RETRACTED

**Figure 1:** Association of PP4R2 and PP4C with phospho-IKK correlates with decline in IKK/NF-κB signaling, COX-2 and Snail in the late phase of PGE2 stimulation **A** and **B.** Lung cancer cells (A549) were treated with PGE2 (20 μg/ml) for various durations and the proteins of the treated cells were examined by immunoblotting as indicated. **C.** The cell extracts were immunoprecipitated with anti-phospho-IKKα/β^S176/180^ or control IgGs antibodies and the pull-down proteins were detected by immunoblotting. β–actin was used as a loading control. Blots are representative of three independent experiments.

### PP4R2/PP4C suppresses IKK phosphorylation

Signal mediators or effectors are known to be dephosphorylated by phosphatases [7]. We thus co-immunoprecipitated phospho-IKKα/β^S176/180^ with several potential phosphatase candidates to examine whether any of the phosphatases can bind and dephosphorylate phospho-IKKα/β^S176/180^ during the late phase of PGE2 or growth factor stimulation. Our results showed that during the late phase, PP4C but not PP1, PP2A or PP5 co-immunoprecipitated with phospho-IKKα/β^S176/180^ (Figure 1C). As PP4C is known to be activated by PP4R1, PP4R2, PP4R3α/β or PP4R4, that may form a holoenzyme with PP4C to increase its binding to the target molecules [14, 15], we also evaluated whether PP4R1, PP4R2, PP4R3α/β or PP4R4 could co-immunoprecipitate with phospho-IKKα/β^S176/180^. Our results showed that there was an increase in PP4R2 but not PP4R1 co-immunoprecipitated with phospho-IKKα/β^S176/180^ during the late phase, whereas PP4 R3α/β and PP4R4 did not interact with phospho-IKKα/β^S176/180^ in lung cancer cells (Figure 1C). In addition, there was more PP4R2 but not PP4R1 co-immunoprecipitated with PP4C (Supplementary Figure S2A). PP4R2 by itself did not dephosphorylate IKK (Supplementary Figure S2B); PP4C caused slight dephosphorylation of IKK and this dephosphorylating effect of PP4C was increased dramatically in the presence of PP4R2 (Supplementary Figure S2B).

RETRACTED

We then examined whether or not downregulation of PP4C and PP4R2 increases the level of phosphorylated IKK and NF-κB. Our results revealed that selective downregulation of PP4C decreased IκBα and increased not only the levels of phospho-IKKα/β^S176/180^ and phospho-NF-κB p65^S536^ but also COX-2 and Snail in the late phase of PGE2 stimulation (Supplementary Figure S3A and S3B; right panels). Interestingly, although knockdown of PP4C downregulated cellular PP4C activity, it did not affect the amount of PP4R2 co-immunoprecipitated with phospho-IKKα/β^S176/180^ (Supplementary Figure S3C; right panels). Knockdown of PP4R2 decreased IκBα and enhanced phospho-IKKα/β^S176/180^, phospho-NF-κB p65^S536^, COX-2 as well as Snail in the late phase of PGE2 stimulation (Figure 2A and 2B; left panels). It also abolished the association of PP4C with phospho-IKKα/β^S176/180^ (Figure 2C; left panels). Unlike knockdown of PP4C and PP4R2, downregulation of control siRNA (Supplementary Figure S3) or PP4R1 (Figure 2A, 2B, 2C; right panels) did not show significant effects on phospho-IKKα/β^S176/180^, phospho-NF-κB p65^S536^, COX-2 and Snail.

**Figure 2:** Knockdown of PP4R2 decreases the association of PP4C to phospho-IKK and enhances IKK/NF-κB signaling, COX-2 and Snail Lung cancer cells (A549) were transfected with PP4R2 siRNA (*siPP4R2*) or PP4R1 siRNA (*siPP4R1*) for 48 h and then treated with PGE2 (20 μg/mL) for various durations as indicated. **A** and **B.** Cells were examined by immunoblotting for protein expression. **C.** The cell extracts were immunoprecipitated with anti-phospho-IKKα/β^S176/180^ or control IgGs antibodies, and the pull-down proteins were detected by immunoblotting (top panel).

### PATZ1 increases PP4R2 expression

To find out what factor(s) might bind to the promoter region of *PP4R2* gene to enhance PP4R2 expression, we searched the TRANSFAC [16] and DECODE (SABiosciences, Frederick, MD, USA) databases. Both databases indicated that PATZ1 would be the most likely candidate. Since PATZ1 is known to exist as four alternatively spliced transcript variants with distinct C-terminal sequences and different molecular weights (74, 69, 58 and 57 kd), respectively, we used polyclonal antibodies (H-300, Santa Cruz Biotechnology) that interacted mainly with the conserved N-terminal domains to detect all 4 variants of PATZ1. We found that the antibodies detected primarily 2 bands i.e., 74 kd (variant 1) and 57 kd (variant 4) PATZ1 in lung cancer cells (Supplementary Figure S1). During sustained stimulation of growth factors, only variant 4 was increased in a time dependent manner (Supplementary Figure S1). We have thus concentrated on studying PATZ1 variant 4 instead of other variants in the subsequent experiments.

RETRACTED

Immunoblotting of lung cancer cells showed that 6 h after PGE2 stimulation PATZ1 (variant 4) started to increase, reaching a plateau level at 24 h and then declining (Figure 3A). The increase of PATZ1 was about 6 h before the increase of PP4R2 that occurred at 12 h after PGE2 stimulation (Figure 3A and Supplementary Figure S2). Unlike PP4R2, neither PP4R3α/β nor PP4R4 was increased after appearance of PATZ1 during sustained stimulation with PGE2 and growth factors (Supplementary Figure S1). Firefly and Renilla dual luciferase reporter assay showed that PATZ1 plasmid (*pPATZ1*) increased PP4R2 gene transcription in a dose-dependent manner (Supplementary Figure S4A) and knockdown of PATZ1 reversed PIP3-stimulated PP4R2 gene transcription (Supplementary Figure S4B). To verify these observations and to assess the interactions of PATZ1 protein with the PP4R2 promoter we performed chromatin immunoprecipitation (ChIP) assay. An increase of the association of PATZ1 protein with the PP4R2 gene at about +363 of transcription start site region was observed in PIP3-treated A549 and CL1-5 lung cancer cells (Supplementary Figure S4C), indicating that PIP3 induces PATZ1 that directly binds to the promoter region of PP4R2 gene and turns on PP4R2 transcription. The induction of PATZ1 was phospho-IKK dependent as downregulation of IKK with dominant negative IKK resulted in a decline of not only phospho-NF-κB p65^S536^ but also PATZ1 and PP4R2 (Figure 3B). Knockdown of PATZ1 abolished the PGE2-mediated induction of PP4R2 leading to sustained high levels of phospho-IKKα/β^S176/180^ and phospho-NF-κB p65^S536^ in the late phase of PGE-2 stimulation (Figure 3C; right panel). Interestingly, PATZ1 knockdown did not affect the levels of PP4C and PP4R1 (Figure 3C; left panel), suggesting that the decrease of phospho-IKKα/β^S176/180^ and phospho-NF-κB p65^S536^, in the late phase is primary due to PATZ1-mediated increase in PP4R2 rather than PP4C.

**Figure 3:** Knockdown of PATZ1 decreases PP4R2 but not PP4C and increases IKK/IkB/NF-kB signaling in the late phase of PGE2 stimulation Lung cancer cells (A549) were transfected with **A.** Control scrambled siRNA (*siCont*), **B.** Empty vector, wild type IKK, dominant negative IKK and **C.** PATZ1 siRNA (*siPATZ1*) for 48 h and then treated with PGE2 (20 μg/mL) for various durations as indicated. Cells were examined by immunoblotting for protein expression.

RETRACTED

### PATZ1 and PP4R2 suppress migration/metastasis

We also examined the effects of PATZ1, PP4R2 and PP4C on matrix metalloproteinases (MMPs) and the migration/invasion of lung cancer cells. Our results showed that MMP-2 and migration/invasion of all 4 lung cancer cell lines i.e., A549, H1299, CL1-0 and CL1-5 were increased by knockdown of PP4R2, PP4C or PATZ1 but not PP4R1 (Supplementary Figure S5 and S6). Overexpression of PATZ1, PP4R2 or PP4C, on the other hand, decreased MMP-2 and migration/invasion of lung cancer cells (Figure 4 and Supplementary Figure S7). Moreover, all the effects of growth factors (EGF, HGF, and IGF-1) and PGE2 on phospho-IKKα/β^S176/180^, phospho-NF-κB p65^S536^, COX-2, Snail as well as epithelial-mesenchymal transition, MMP-2 and migration/invasion of the lung cancer were attenuated by upregulation of PATZ1 (Figure 4). To further verify the critical role of PP4R2/PP4C in the effects of PATZ1, we overexpressed PATZ1 and then downregulated PP4R1, PP4R2 or PP4C. Our results showed that PATZ1-mediated decrease in IKK/NF-κB signaling, COX-2, Snail, MMP-2 activity and migration/invasion of lung cancer cells was restored by downregulating PP4R2 and PP4C but not PP4R1 (Supplementary Figure S8).

**Figure 4:** Overexpression of PATZ1 attenuates the effects of growth factors and PGE2 on phospho-NF-κB, COX-2, Snail, EMT and MMP-2 activity as well as migration/invasion of the lung cancer cells Lung cancer cells (A549 and CL1-5) were transfected either with control empty vector (EV) or pCMV6-*PATZ1* (*pPATZ1*) for 24 h and then treated for 24 h with 20 μg/ml of PGE2 or 100 ng/ml growth factors as indicated. **A.** The cell lysates were examined by immunoblotting for protein expression. PATZ1, phospho-IKKα/β^S176/180^, IKKα/β, phospho-NF-κB p65^S536^ and NF-κB were measured at 1 h, all the others were determined at 24 h after PGE2 and growth factor treatment. **B** and **C.** The migration and invasion abilities of cells were examined by transwell assays after 20 h incubation. The activities of MMP-2 in cell-conditioned media were analyzed by gelatin zymography after culturing cells in serum-free medium for 24 h. Blots are representative of three independent experiments. Data represent means ± s.d. of three independent experiments; *P < 0.05 by t-test.

In addition, we examined the IHC staining of PATZ1 and PP4R2 in matched pairs of lung carcinoma tissue specimens from primary lung tumors and lymph node metastases. Our results showed that the median levels of PATZ1 and PP4R2 were higher in primary tumors versus lymph node metastases of the patients (n = 80; *P* < 0.001) (Figure 5A). Both adenocarcinoma (ADC, n = 34; *P* < 0.001) and squamous cell carcinoma (SCC, n = 34; *P* < 0.001) showed similar results (Figure 5B). Moreover, the metastatic tumors with lower PATZ1 also tended to exhibit lower PP4R2 (Pearson correlation = 0.71, *P* < 0.0001; Figure 5C).

RETRACTED

**Figure 5:** Lung cancers at the primary sites have more PP4R2 and PATZ1 than those at the metastatic sites Lung tissue sections from human lung carcinoma microarrays were immunostained with anti-PATZ1 and anti-PP4R2 antibodies, respectively. **A** and **B.** The PATZ1 and PP4R2 level in matched pairs of tumor tissues specimens were scored according to the percentage and intensity of positive cells. More PATZ1 and PP4R2 were found in primary than lymph node metastases lung carcinoma. Data are expressed as medians relative to each group of tissues. ***P < 0.001. **C.** Scatter plot was generated by plotting the levels of PATZ1 versus those of PP4R2 (left panel; Pearson correlation = 0.71, P < 0.0001). The representative lung tumor sections were examined at ×200 magnification for PATZ1 and PP4R2 (right panel). Scale bar is 100 μm.

To investigate whether ectopic PATZ1 or PP4R2 is sufficient to suppress lung cancer colonization/metastasis *in vivo*, we generated A549^GL^, A549^EV-GL^, A549^shCont-GL^, A549^pPATZ1-GL^, A549^pPP4R2-GL^, A549^shPP4R2-1-GL^, A549^shPP4R2-2-GL^, A549^pPATZ1/shPP4R2-1-GL^, or A549^pPATZ1/shPP4R2-2-GL^ cells, stably expressing not only green fluorescent protein and luciferase (GL) but also empty vector (EV), control shRNA (shCont), PATZ1 (pPATZ1), PP4R2 (pPP4R2), PP4R2 shRNA (shPP4R2-1 or shPP4R2-2), or PATZ1 cDNA and shPP4R2 (pPATZ1/shPP4R2-1 or pPATZ1/shPP4R2-2) as indicated (Figure 6A). *In vitro* cell proliferation assay for 3 days revealed that the proliferation rate of the cells overexpressing PATZ1 and PP4R2 (i.e., A549^pPATZ1-GL^ and A549^pPP4R2-GL^) was lower than the remaining groups (Figure 6B). Examination of 3-dimensional growth and MMP-2 activity showed that cells overexpressing either PATZ1 or PP4R2 formed fewer colonies and produced less MMP-2 activity, whereas cells with downregulation of PP4R2 (i.e., A549^shPP4R2-1-GL^ and A549^shPP4R2-2-GL^) had more colonies and MMP-2 activity than the other cells (Figure 6C). Likewise, A549^pPATZ1-GL^ and A549^pPP4R2-GL^ cells exhibited less, whereas A549^shPP4R2-1-GL^ and A549^shPP4R2-2-GL^ cells exhibited more migration/invasion ability than the others (Figure 6D).

RETRACTED

**Figure 6:** PATZ1 and PP4R2 suppress 3-dimensional growth and invasive ability of lung cancer cells *in vitro* A549^GL^, A549^EV-GL^, A549^shCont-GL^, A549^pPATZ1-GL^, A549^pPP4R2-GL^, A549^shPP4R2-1-GL^, A549^shPP4R2-2-GL^, A549^pPATZ1/shPP4R2-1-GL^, and A549^pPATZ1/shPP4R2-2-GL^ cells were generated. **A.** Cells were examined by immunoblotting for protein expression. Blots are representative of 3 independent experiments. **B.** Growth of cells was examined by BrdU cell proliferation assay. **C.** Anchorage-independent growth and MMP2 enzyme activity of cells were examined by soft agar assay and gelatin zymography assay. **D.** Migration and invasion of cells were examined by transwell assay. Data represent means ± s.d. of 3 independent experiments; *P < 0.05 by one-way ANOVA.

Inoculation of mice with these cells demonstrated that on day 49 post-inoculation mice bearing cancer cells overexpressing PATZ1 or PP4R2 (A549^pPATZ1-GL^ or A549^pPP4R2-GL^) developed the least whereas, those bearing cancer cells with downregulation of PP4R2 (A549^shPP4R2-1-GL^ or A549^shPP4R2-2-GL^) developed the most tumor nodules (Figure 7A and 7B). Downregulation of PP4R2 in cancer cells overexpressing PATZ1 (A549^pPATZ1/shPP4R2-1-GL^ and A549^pPATZ1/shPP4R2-2-GL^) resulted in the development of about the same number of tumor nodules as mice bearing A549^GL^, A549^EV-GL^ or A549^shCont-GL^ cells (Figure 7A and 7B). Immunoblot analysis of the lung tissue lysates showed that mice bearing cancer cells overexpressing PATZ1 or PP4R2 (A549^pPATZ1-GL^ or A549^pPP4R2-GL^) had the lowest levels of phospho-IKKα/β^S176/180^, phospho-NF-κB p65^S536^, COX-2, Snail and EMT (Figure 7C). In comparison, mice bearing cancer cells with downregulation of PP4R2 (A549^shPP4R2-1-GL^ or A549^shPP4R2-2-GL^) developed the highest levels of phospho-IKKα/β^S176/180^, phospho-NF-κB p65^S536^, COX-2, Snail and EMT (Figure 7C). Immunohistochemical examination of lung tissue sections revealed that there was less proliferation (as indicated by Ki67 index) and more upregulation of E-cadherin in tumors of the mice bearing A549^pPP4R2-GL^ and A549^pPATZ1-GL^ cells than in tumors of those bearing A549^EV-GL^, A549^shCont-GL^, A549^pPATZ1/shPP4R2-1-GL^, A549^pPATZ1/shPP4R2-2-GL^, 549^shPP4R2-1-GL^ or A549^shPP4R2-2-GL^ cells (Figure 7D). Moreover, all the mice bearing cancer cells with downregulation of PP4R2 (A549^shPP4R2-1-GL^ or A549^shPP4R2-2-GL^) had median survival time of 47 days post inoculation that was 16 days earlier than mice bearing A549^GL^, A549^EV-GL^ and A549^shCont-GL^ (Figure 7E). In contrast, the mice bearing cancer cells overexpressing PATZ1 or PP4R2 (A549^pPATZ1-GL^ or A549^pPP4R2-GL^) had median survival time of 96 days (Figure 7E). Knockdown of PP4R2 in cells overexpressing PATZ1 (A549^pPATZ1/shPP4R2-1-GL^ and A549^pPATZ1/shPP4R2-2-GL^) resulted in decrease of median survival time to around 68 days post-inoculation (Figure 7E).

RETRACTED

**Figure 7:** PATZ1 and PP4R2 suppress lung cancer metastasis *in vivo* The cells were injected respectively into tail veins of 9 groups of mice (1 × 10^6^/50 μl/mouse) in the order as indicated in Figure 6A. **A.** The whole bodies of mice were detected by bioluminescent imaging. **B.** The lungs of 3 mice in each group were dissected from the surrounding tissue for tumor nodule measurement. **C.** Cell lysates of 3 lung tissue samples from 3 mice in each group were extracted and analyzed by immunoblotting respectively. Blots are representative of 3 independent experiments. **D.** The murine lung sections were analyzed after H&E (×100 magnification) and immunohistochemistry staining (×100 magnification). Data represent means ± s.d.; *P < 0.05 by one-way ANOVA. Scale bar is 100 μm. **E.** Comparison of life span showed that mice inoculated with A549^pPATZ1-GL^ or A549^pPP4R2-GL^ cells had the longest lifespan (> 84 days; *P* < 0.001, *n* = 6 by one-way ANOVA) in all A549 xenograft mice.

## DISCUSSION

Brechmann and coworkers reported previously that PP4R1 bridges the IKK complex and the phosphatase PP4C, thereby dephosphorylating and inactivating the IKK complex in a subgroup of T cell lymphomas and polyclonal mitogen PHA-stimulated human T lymphocytes [14]. However, they did not elucidate how PP4R1 transcription was increased and explore whether or not other PP4 regulatory subunit(s) such as PP4R2 have a similar effect to PP4R1 in T cell lymphomas or other cancers. Here, we found that PP4R2 rather than PP4R1was increased in a variety of lung cancer cells under growth factor or PGE2 stimulation (Figure 1, 2 and Supplementary Figure S1, S2, and S3). The transcription of PP4R2 in lung cancer was selectively enhanced by transcriptional factor PATZ1 variant 4 that binds to the promoter region of the *PP4R2* gene (Figure 3A and Supplementary Figure S4). Ectopic PP4R2 but not PP4R1 decreased phosphorylated IKK/NF-κB, EMT, MMP-2 and migration/invasion of lung cancer (Supplementary Figure S7). How PP4R1 and PP4R2 show distinct effects on phospho-IKK in different cancer types under different stimuli remains to be elucidated.

Ectopic PATZ1 has recently been shown by Chiappetta and coworkers to suppress thyroid cancer migration/invasion [17]. Since PATZ1 may regulate transcription of p53-target genes [12, 18], Chiappetta and coworkers proposed that the inhibitory effects of PATZ1 could be due to p53-dependent motility-related genes in three thyroid cancer cell lines [17]. However, they found that the p53-dependent genes exhibited distinct responsiveness to PATZ1 in different thyroid cell lines. They thus suggested that further experiments are needed to better elucidate the dynamics of PATZ1 binding to these genes in relation to the presence/absence of a functional p53 protein. Here, we found that PATZ1 and PP4R2 were consistently increased after sustained PIP3, PGE2 or growth factor stimulation and were phospho-IKK dependent (Supplementary Figures S1, S2A, and Figure 3A and 3B). PATZ1-induced PP4R2 was positively associated not only with inactivation of phospho-IKK but also inhibition of migration/invasion of lung cancer cells regardless of whether the lung cancer cells express wild p53 (A549), p53 null (H1299) or p53 mutant (CL1-0 and CL1-5) (Figure 3 and Supplementary Figures S5-S8). The median levels of PATZ1 and PP4R2 were higher in primary tumors versus lymph node metastases in patients (n = 80; *P* < 0.001) (Figure 5A). In addition, mice inoculated with A549 mutant cells that overexpressed PATZ1 or PP4R2 (A549^pPATZ1-GL^ or A549^pPP4R2-GL^) had the lowest level of phospho-IKK and phospho-NF-κB in their tumors (Figure 7C) as well as the longest lifespan (Figure 7E; median survival time of 96 days vs 63 days; *P* < 0.001, *n* = 6 by one-way ANOVA), whereas, PP4R2 knockdown suppressed not only PP4R2 but also the level of PATZ1, reversed the inhibitory effects of PATZ1 on phosphorylation of IKK and NF-κB and shortened the lifespan of xenograft mice (Figure 7). These results unravel the existence of a negative feedback loop of PATZ1 and PP4R2 on IKK/NF-κB signaling, that suppresses lung cancer migration/invasion capability (Figure 8).

RETRACTED

**Figure 8:** Schematic diagram illustrates the roles of PATZ-1 and PP4R2 in regulating the effects of growth factors and PGE2 on IKK/NF-κB signaling, COX-2, Snail and migration/invasion of lung cancer

How can cancer cells form a visible size of primary tumor and then metastasize to distant tissues is still not well understood. Our results suggest that the presence of PATZ1 and PP4R2 negative feedback loop on IKK/NF-κB signaling as depicted in Figure 8 may prevent cancer cells from over-stimulation from growth factors or inflammatory mediators so that they can postpone early dissemination and accumulate to form visible or even massive size of primary tumors to decrease the chance of being individually destroyed by immune cells. When the mutant cells with lower level of PATZ1 and PP4R2 emerge in late stages of tumor progression, they would then have more capability for migration/invasion and be able to metastasize to the distant tissues (Figures 5, 7A, 7B). Our uncovering of PATZ1 and PP4R2 negative feedback loop, on the other hand, may facilitate the design of novel approaches for clinical interventions at different stages in disorders induced by aberrant elevation of active IKK/NF-κB signaling.

## MATERIALS AND METHODS

### Reagents

The materials were purchased and obtained as follows: Recombinant human EGF, HGF and IGF-1 were from R&D Systems (Abingdon, UK); pCMV6-*PP4R1* (NM_005134), pCMV6-*PP4R2* (NM_174907), pCMV6*-PP4C* (NM_002720), pCMV6*-PATZ1 variant 3* (NM_032052), and pCMV6*-PATZ1 variant 4* (NM_032051) plasmids were from ORIGENE (Rockville, MD); *PATZ1 variant 4* and *PP4R2* genes from pCMV6-*PATZ1* and pCMV6-*PP4R2* plasmids subcloned into pCMV6-AC-mCFP plasmids (ORIGENE) were applied for the establishment of PATZ1- and PP4R2-transduced stable cells. pCMV2-IKKβ WT (wild type; WT), pCMV2-IKKβ S177ES181E (dominant active; DA) and pCMV2-IKKβ K44M (dominant negative; DN) were obtained from Addgene (Cambridge, MA; plasmid numbers 11103 and 11104) and were originally created by Dr. Anjana Rao laboratory. control siRNAs, PP4R1-siRNA, PP4R2-siRNA, PP4C-siRNA and PATZ1-siRNA were all from Santa Cruz Biotechnology (Santa Cruz, CA); two shRNA HuSH 29mer shRNA (TF302311A and TF302311C) constructs against PP4R2 in pRFP-C-RS vector and the non-effective 29-mer scrambled shRNA (TR30015) were from ORIGENE; mouse anti-Vimentin (V9) antibodies and recombinant PGE2 were from Sigma-Aldrich (St Louis, MO); phosphatidylinositol (3,4,5)-trisphosphate diC16 (PI(3,4,5)P3 diC16) were from Echelon Biosciences (Salt Lake City, UT); Anti-PP4R1 (ab70624), anti-PP4R2 (ab70631), anti-PP4C (ab16475), anti-PP4R3α (ab70635), anti-PP4R3β (ab70622), anti-PP4R4 (ab111419), and anti-PATZ1 (ab154025) rabbit polyclonal antibodies were from Abcam (Cambridge, UK); mouse anti-PP1 (E-9), mouse anti-PP5 (H-7), rabbit anti-PHB (H-80), rabbit anti-IKKα/β (H-470), mouse anti-β-actin (C-4), goat anti-COX-2 (M-19), rabbit anti-E-cadherin (H-108), rabbit anti-ZEB1 (H-102), rabbit anti-Snail (H-130), rabbit anti-Twist (H-81), and rabbit anti-PATZ1 (H-300) antibodies as well as horseradish peroxidase-conjugated anti-mouse IgG, horseradish peroxidase-conjugated anti-goat IgG and horseradish peroxidase-conjugated anti-rabbit IgG antibodies were from Santa Cruz Biotechnology (Santa Cruz, CA); rabbit anti-PI3Kp85, rabbit anti-PI3Kp85^Y458^, rabbit anti-Akt, rabbit anti-phospho-Akt^Ser473^, rabbit anti-phospho-IKKα/β^S176/S180^ and rabbit anti-phospho-NF-κBp65^S536^, horseradish peroxidase-conjugated mouse-anti-rabbit IgG (Conformation Specific; L27A9) antibodies were from Cell Signaling Technology (Beverly, MA); and rabbit anti-IκB, rabbit anti-NF-κBp65 and rabbit anti-Raf-1 antibodies were from Millipore (Temecula, CA).

RETRACTED

### Cell culture

A549 cell line (ATCC: CCL-185), H1299 (ATCC: CRL-5803), CL1-0 and CL1-5 cells [19, 20] were maintained in DMEM or RPMI medium (GibcoBRL Life Technologies, Grand Island, NY) supplemented with 10% fetal bovine serum (FBS; GibcoBRL Life Technologies) and 1% penicillin-streptomycin-neomycin (GibcoBRL Life Technologies). Unless otherwise specified, 2 × 10^5^/mL cells were used in each experiment. A549 and H1299 cells were obtained directly from the cell bank of Food Industry Research and Development Institute (Hsinchu, Taiwan). The cell lines were certified by the Food Industry Research and Development Institute (Hsinchu, Taiwan) using STR-PCR method and passaged in our laboratory for fewer than 6 months after resuscitation. A549 has wild-type p53; H1299 is p53 null [21] whereas CL1-0 and CL1-5 are p53 mutated (p53^R248W^) [20]. *In vitro* cell viability was measured by WST-1 assay according to the manufacturer's instructions (Roche, Mannheim, Germany) and cell proliferation was determined by BrdU (5-bromo-2′-deoxyuridine) cell proliferation ELISA kit (Abcam).

### Transfection of cDNA, siRNAs and shRNA

cDNA, siRNAs and shRNA were transfected into cell lines by GenMute siRNA Transfection Reagent (SignaGen Laboratories, Gaithersburg, MD) according to the manufacturer's protocol. The expression of target proteins in the transfected cells was determined 48 h after transfection, unless specified otherwise. The cDNA- or shRNA-transduced cells were selected by G418 or puromycin (Sigma-Aldrich, St. Louis, MO).

### Immunoblotting, immunoprecipitation and gelatin zymographic analysis

Gelatinolytic activities of MMP-2 and MMP-9, immunoprecipitation and immunoblotting were performed as described previously [22, 23]. Briefly, supernatants were collected and concentrated with Vivaspin 6 centrifugal concentrators (Vivascience, VS2002) for zymographic analysis. Twenty micrograms of concentrated supernatants were loaded for electrophoresis under nonreducing conditions on 10% SDS-polyacrylamide gels containing 1 mg/ml gelatin. After electrophoresis, the gels were washed in 2.5% Triton X-100 and then incubated for 20 h at 37°C in the development buffer containing 0.01 M CaCl_2_, 0.05 M Tris-HCl (pH 8.0). The zymographic gels were fixed in 50% Coomassie brilliant blue R-250, then destained in 10% acetic acid. The bands were quantified with ImageQuant 5.2 software (Amershan Bioscience).

### Migration, invasion assays and anchorage-independent growth assays

Migration, invasion and anchorage-independent growth assays were performed *in vitro* as described previously [6, 24]. Briefly, transwell inserts (8 μm pore; Costar, 3422) were placed into the wells for cell migration assay. A total of 2 × 10^4^ cells in serum free-medium were placed in the upper chamber and 10% FBS-medium were placed in the lower chamber. After incubation at 37°C in a humidified 5% CO_2_ atmosphere for 20 h, the cells that had migrated to another side of membrane were fixed with methanol and the non-migrated cells were mechanically removed with a cotton swab. Cells adherent on the membrane were stained with Liu's stain (ASK, 03R011/03R021). Cell numbers were examined under light microscopy at 200 × magnification. For cell invasion assay, the process was similar as migration assay except that matrigel had been thawed and liquefied on ice, and then 50 μl of matrigel was added to a transwell insert and solidified in a 37°C incubator to form a thin gel layer before application of cells. As to anchorage-independent growth assay, 1 × 10^3^ cells were suspended in 0.33% Bacto agar (Sigma-Aldrich) mixed with 10% FBS and antibiotics in DMEM. Suspended cells were layered over 0.5% Bacto agar in the same medium in a 60-mm dish. On day 21, cells were fixed and stained for the examination of colony growth, colonies > 60 μm (> 60 cells) were counted and results were expressed as the mean number of colonies ± s.d.

RETRACTED

### Phosphatase assay

To determine dephosphorylation of phospho-IKK by PP4R2 and PP4C *in vitro*, Myc: PP4R2, Myc:PP4C or Flag:phospho-IKKβ were isolated with Pierce Direct IP kit (Thermo SCIENTIFIC, Rockford, IL) from Myc:PP4R2-, Myc:PP4C- and Flag:DA-IKKβ-transfected CL1-0 cells, respectively. Equivalent portion of these isolated proteins were co-incubated for 30 min at 37°C in phosphatase buffer (50 mM Tris-HCl, PH7.0, 0.1 mM CaCl2, 0.1 mg/ml bovine serum albumin (BSA) and 1mM MnCl_2_). IKK phosphorylation and dephosphorylation were then assessed by immunoblotting. To measure phosphatase activity of endogenous of PP4C, cells were washed in TBS and then lysed on ice in phosphatase assay buffer (20 mM imidazole-HCl, 2 mM EDTA, 2 mM EGTA, and 0.1% NP-40, pH 7.0) with freshly added protease inhibitors. PP4C was immunoprecipitated out after mixing 1 mg of total cell lysates with 3 μg of anti-PP4C antibodies (ab16475, Abcam) and Protein G agarose for 2 h at 4°C. PP4C activity was assayed by incubating the immunoprecipitated protein with the synthetic phosphopeptide K-R-pT-I-R-R at 30°C for 10 min prior to detection with malachite green phosphate detection solution, according to the manufacturer's instructions (cat: 17-313, Millipore). Phosphatase activity was normalized to the relative amount of untreated control cells according to western blot quantitation as indicated.

RETRACTED

### Luciferase reporter assay

To examine transcriptional regulation of PP4R2 gene promoter, approximately 3 kb of the *PP4R2* promoter (−2500/+500) was synthesized by GenScript (Genscript Corporation, Piscataway, NJ) and subcloned into the pGL3-basic vector (Promega, Madison, WI) to generate the *PP4R2* promoter/firefly luciferase reporter construct, designated pGL3-*PP4R2*. pRL-TK plasmid (Promega) containing *Renilla* luciferase was used as an internal control. At 24-36 h after transfection, cell lysates were assayed using the Dual-Luciferase Reporter Assay System (Promega) and luciferase activities were measured with a luminometer (Wallac Vector3; PerkinElmer, Boston, MA) in the same manner as described previously [6].

### Chromatin immunoprecipitation assay

Chromatin immunoprecipitation (ChIP) assays were performed according to the manufacturer's protocol (EZ–Magna ChIP A/G kit; Millipore, Billerica, MA). Cells were incubated for 12 h with PIP3 or medium alone before cross-linking protein complexes to DNA using 1% formaldehyde (Sigma-Aldrich). Samples were sonicated on ice (Ultrasonic Disruptor UD-201; TOMY, Tokyo, Japan) to generate 200-1000 DNA fragments. DNA was incubated with Protein A/G magnetic beads alone or with beads plus anti-PATZ1 (H-300; Santa Cruz Biotechnology) or IgG isotype control antibodies. The beads were pelleted with a magnetic separator and purified DNA was analyzed by SYBR green real time PCR using EpiTect ChIP qPCR Assay (Qiagen, Valencia, CA) with specific primers against the proximal region of human pp4r2 gene promoter (GPH1009388(+)01A; +363 bp from the transcription start site). Data are expressed as percentage relative to the untreated control.

### Preparation of pCMV-GFP/luciferase-lentivirus and establishment of stable cell lines

A549^GL^ cells were produced by infecting A549 cells with cytomegalovirus promoter (pCMV)-GFP/luciferase-lentivirus as described previously [6]. A549^GL^ cell lines were transfected with empty vector (EV), control shRNA (shCont), PATZ1 (pPATZ1), PP4R2 (pPP4R2), PP4R2 shRNA (shPP4R2-1 or shPP4R2-2), or PATZ1 and shPP4R2 (PATZ1/shPP4R2-1 or PATZ1/shPP4R2-2) separately and selected with G418 (400 μg/mL) or Puromycin (1 μg/mL) to produce A549^EV-GL^, A549^shCont-GL^, A549^pPATZ1-GL^, A549^pPP4R2-GL^, A549^shPP4R2-1-GL^, A549^shPP4R2-2-GL^, A549^pPATZ1/shPP4R2-1-GL^, or A549^pPATZ1/shPP4R2-2-GL^. The expression levels and effects of PATZ1 and PP4R2 shRNA in each stable cell line were examined by immunoblotting, cell proliferation assay, anchorage-independent growth assay, gelatin zymography assay, migration and invasion assays *in vitro*.

RETRACTED

### Experimental xenograft murine metastasis model

Male severe combined immunodeficiency (SCID) mice (C.B17/lcr-Prkdc ^scid^/CrlNarl) were purchased from the National Laboratory Animal Center (Taipei, Taiwan). All animal care and *in vivo* experiments were performed in compliance with the guidelines of the Academia Sinica Institutional Animal Care and Utilization Committee. Mice (*n* = 9/group) were implanted on day 0 by lateral tail vein injection in the order (1) vehicle, (2) A549^EV-GL^, (3) A549^shCont-GL^, (4) A549^pPATZ1-GL^, (5) A549^pPP4R2-GL^, (6) A549^shPP4R2-1-GL^, (7) A549^shPP4R2-2-GL^ and (8) A549^pPATZ1/shPP4R2-1-GL^ (9) A549^pPATZ1/shPP4R2-2-GL^ cells. Metastatic progression was monitored weekly and quantified using a noninvasive bioluminescence IVIS Imaging System (Xenogen, Alameda, CA) as described previously [6]. Forty-nine days (seven weeks) after injection, three mice were killed for necropsy, H&E, immunohistochemical staining and cell lysate analysis of lung. The other 6 mice were kept to obtain further bioluminescent images of whole body and for survival studies. The percentage of animal survival in each group was routinely recorded.

### Immunohistochemistry and histopathology examination

Human lung cancer tissue microarray slides with matched metastatic lymph node were purchased from US Biomax (LC814a and LC817). Immunohistochemistry and histopathology analyses as well as immunohistochemical scoring were performed in the same manner as described previously [5, 6]. Scores were generated by the percentage of positive cells multiplied by stain intensity (score 0 = negative, 1-2 = weak, 3-4 = moderate, 5-6 = strong). The images were scanned into a digital format by Scanscope XT system (Aperio Technologies, Vista, CA) and analyzed using Aperio ImageScope 9.1 software (Aperio Technologies).

### Statistics

The survival time was assessed using Kaplan-Meier curves and tested for significance by the log-rank test. Statistical evaluation was performed using GraphPad Prism version 5.0 for Microsoft Windows (GraphPad Software, La Jolla, CA). Differences among multiple groups of data were analyzed by one-way ANOVA followed by a multiple comparisons test. Differences between groups were considered statistically significant at P values of less than 0.05 or 0.01.

## SUPPLEMENTARY FIGURES


